# Intelligent Deep Learning Enabled Oral Squamous Cell Carcinoma Detection and Classification Using Biomedical Images

**DOI:** 10.1155/2022/7643967

**Published:** 2022-06-30

**Authors:** Adwan A. Alanazi, Manal M. Khayyat, Mashael M. Khayyat, Bushra M. Elamin Elnaim, Sayed Abdel-Khalek

**Affiliations:** ^1^Department of Computer Science and Information, University of Hail, Hail, Saudi Arabia; ^2^Department of Information Systems, College of Computers and Information Systems, Umm Al-Qura University, Makkah, Saudi Arabia; ^3^Department of Information Systems and Technology, College of Computer Science and Engineering, University of Jeddah, Jeddah, Saudi Arabia; ^4^Department of Computer Science College of Science and Humanities in Al-Sulail, Prince Sattam Bin Abdulaziz University, Al-Kharj, Saudi Arabia; ^5^Department of Mathematics and Statistics, College of Science, Taif University, P. O Box 11099, Taif 21944, Saudi Arabia

## Abstract

Oral cancer is one of the lethal diseases among the available malignant tumors globally, and it has become a challenging health issue in developing and low-to-middle income countries. The prognosis of oral cancer remains poor because over 50% of patients are recognized at advanced stages. Earlier detection and screening models for oral cancer are mainly based on experts' knowledge, and it necessitates an automated tool for oral cancer detection. The recent developments of computational intelligence (CI) and computer vision-based approaches help to accomplish enhanced performance in medical-image-related tasks. This article develops an intelligent deep learning enabled oral squamous cell carcinoma detection and classification (IDL-OSCDC) technique using biomedical images. The presented IDL-OSCDC model involves the recognition and classification of oral cancer on biomedical images. The proposed IDL-OSCDC model employs Gabor filtering (GF) as a preprocessing step to eliminate noise content. In addition, the NasNet model is exploited for the generation of high-level deep features from the input images. Moreover, an enhanced grasshopper optimization algorithm (EGOA)-based deep belief network (DBN) model is employed for oral cancer detection and classification. The hyperparameter tuning of the DBN model is performed using the EGOA algorithm which in turn boosts the classification outcomes. The experimentation outcomes of the IDL-OSCDC model using a benchmark biomedical imaging dataset highlighted its promising performance over the other methods with maximum accu_*y*_, prec_*n*_, reca_*l*_, and *F*_score_ of 95%, 96.15%, 93.75%, and 94.67% correspondingly.

## 1. Introduction

Oral cancer is leading cancer globally and is considered by late diagnoses, morbidity higher, and mortality rates. Two-third of the total occurrence arises in low- and middle-income countries (LMICs), and half of the cases are in South Asia [1, 2]. Excessive usage of alcohol and tobacco are the main risk factor for oral tumors. The major factor in South and Southeast Asia is betel quid chewing which usually comprises slaked lime, betel leaf, and areca nut and might comprise tobacco [3]. Currently, they are commercially offered in sachets and are common in public because of their dynamic marketing strategy. The oral lesion is related to late presentation, mainly in LMIC, around two-third present at a late stage, and consequently, the survival rate is poor [4]. Cancer management, particularly at the late stage, is too expensive [5]. The lack of knowledge of health professionals and lack of public awareness concerning oral lesions are major reasons for late diagnosis. The OPMD diagnosis has a risk of malignant transformation, is of great significance to reduce mortality and morbidity from oral tumors, and has been the major emphasis of the screening program [6]. But the application of this program depends on visual inspection has turned out to be challenging in real-time settings as they depend on healthcare professionals, who are not experienced or adequately trained to identify this lesion [7, 8].

Earlier identification of OSCC gains significant importance for improved diagnosis, treatment, and survival [5, 6]. Late diagnosis has hampered the quest for precision medicine in spite of the advancements in the understanding of the molecular mechanism of cancer. Thus, machine learning (ML) and deep learning (DL) models have been employed for improving recognition and thereby reducing cancer-specific death rates and morbidity [7]. Automated image examination clearly has the significance of assisting pathologists and clinicians in the earlier detection of OSCC and decision-making in management. The considerable heterogeneity in the presence of oral cancer makes the detection highly complex for healthcare professionals and common cause of delays in inpatient referral to oral lesion specialists [9]. In addition, early-stage OSCC lesions and OPMD are generally asymptomatic and might seem like small, harmless lesions, leading to late presentation of the patient and eventually leading to diagnosis delay [10, 11]. Advancement in the fields of deep learning and computer vision offers an effective method to propose adjunctive technology that could implement an automatic screening of the oral cavity and present feedback to individuals for self-examination and healthcare professionals at the time of patient examination.

Bhandari et al. [12] aim to improve the performance of classifying and detecting oral tumors within a minimized processing time. The presented technique comprises a convolution neural network with an adapted loss function to minimize the error in classifying and predicting oral tumors by supporting multiclass classification and minimizing the over-fitting of the data. Lu et al. [13] presented an automatic approach for oral tumor diagnosis on slide cytology images. The pipeline comprises per-cell focus selection, CNN-based classification, and fully convolution regression-based nucleus recognition. The proposed method offers faster per-cell focus decisions at human-level accuracy. Song et al. [14] introduced an image classification method based on autofluorescence and white-light images with the DL method. The data are fused, extracted, and calculated to feed the DL-NN. Next, compared and investigated the efficiency of regularization, convolution neural network, and transfer learning technique for classifying oral tumors.

Figueroa et al. [15] designed a DL training model which provides understandability to its prediction and guides the network to remain focused and precisely delineate the tumorous region of the image. Lim et al. [16] developed a DL architecture called D'OraCa to categorize oral lesions with photographic images. It develops a mouth landmark recognition method for the oral image and integrates it with oral cancer classification as guidance to enhance the classification performance. Shamim et al. [17] evaluated and applied the effectiveness of six deep convolutions neural network (DCNN) models with transfer learning, for recognizing precancerous tongue lesions through a smaller data set. DCNN model can distinguish between five kinds of tongue cancer and differentiate between benign and precancerous tongue lesions.

In comparison with conventional ML models, the DL models receive input and do not involve a complicated feature extraction process. Besides, the heterogeneous pattern can result in variance over distinct instances and thereby causes complexity in handcrafted features with restricted generalization ability. In addition, the DL models exhibit high scalability owing to the capability of processing large amounts of data. The considerable heterogeneity in the presence of oral lesions makes the detection process difficult and is considered to be the leading cause of delays in inpatient referrals to oral cancer specialists. In addition, early-stage OSCC lesions remain symptomless and may look like small, inoffensive lesions, resulting in the late demonstration of the patient and eventually leading to additional diagnosis delay. Therefore, it is needed to design effective OSCC classification models.

This article presents an intelligent deep learning enabled oral squamous cell carcinoma detection and classification (IDL-OSCDC) model using biomedical images. The suggested model employs Gabor filtering (GF) as a preprocessing process to eliminate noise content. In addition, the NasNet model is exploited for the generation of high-level deep features from the input images. Moreover, an enhanced grasshopper optimization algorithm (EGOA)-based deep belief network (DBN) model is employed for oral cancer classification and detection. The hyperparameter tuning of the DBN model is performed using the EGOA algorithm which in turn boosts the classification outcomes. The experimentation outcomes of the IDL-OSCDC model are performed using a benchmark biomedical imaging dataset.

The rest of the paper is organized as follows.  Section 2 provides the proposed IDL-OSCDC model, and Section 3 offers the performance validation. At last, Section 4 concludes the study.

## 2. The Proposed IDL-OSCDC Model

In this article, a novel IDL-OSCDC model was introduced for the identification and classification of oral tumors using biomedical images. At the initial stage, the IDL-OSCDC model utilized the GF technique to get rid of noise content. Following this, the NasNet model is exploited for the generation of higher-level deep features from the input images. Finally, the EGOA-DBN model is utilized to detect and categorize oral cancer.  Figure 1 illustrates the overall process of the IDL-OSCDC technique.

### 2.1. Image Preprocessing Using GF Technique

In this study, the IDL-OSCDC model utilized the GF technique to get rid of noise content. The GF is a bandpass filter that is effectively executed for variation of image processing and machine vision application. In 2D, the Gabor function is an oriented complex sinusoidal grating reduced by a 2D Gaussian envelope. In a 2D co-ordinate (*a*, *b*) scheme, the GFs containing real components and imaginary ones are demonstrated as [18]

(1) $$\begin{array}{c} G_{\delta ,\theta ,\psi ,\sigma ,\gamma }\left(a,b\right)=\;\exp\;\left(-\frac{a^{'2}+\gamma^{2}b^{'2}}{2\sigma^{2}}\right)\times \;\exp\;\left(j\left(2\pi \frac{a^{\prime }}{\delta }+\psi \right)\right), \end{array}$$

where

(2) $$\begin{array}{c} a^{\prime }=a\;\cos\;\theta +b\;\sin\;\theta ,\\ b^{\prime }=-a\;\sin\;\theta +b\;\cos\;\theta , \end{array}$$

in which *δ* implies the wavelength of sinusoidal factors, and *θ* signifies the orientation separation angle of the Gabor kernel. Notably, it can be required only to assume *θ* from the interval [0°,  180°] as symmetry creates other directions redundant. *ψ* defines the phase offset, *σ* demonstrates the standard derivation (SD) of the Gaussian envelope, and *γ* denotes the ratio of spatial features (the default value is 0.5) identifying the ellipticity of supports of the Gabor functions. The parameter 0 has been defined by 6 and spatial frequency bandwidth *bw* as

(3) $$\begin{array}{c} \sigma =\frac{\delta }{pi}\sqrt{\frac{\ln2}{2}\;}\frac{2^{bw}+1}{2^{bw}-1}. \end{array}$$

### 2.2. Feature Extraction: NASNet Model

For the effectual derivation of feature vectors, the NASNet model is utilized [19]. The NASNetMobile model is a recently developed DL model with 53,26,716 parameters. It exhibits high reliability. The fundamental component of the NASNet model is the block, and a collection of blocks is integrated to form a cell. The searching space involved in the NASNet is the factorization of the networks to cells and again splits into blocks. The number and type of cells/blocks are not predefined. However, they need to be optimized for the chosen dataset. The probable functioning of the block comprises convolution, separable convolution, max pooling, average pooling, and identify map. The block has the ability of mapping two inputs into an output feature map. It performs element-wise addition. When the cell receives a block with a feature map size of *H* × *W* and stride of 1, the outcome will be the identical size of the feature map.  Figure 2 depicts the framework of the NASNet model.

Once the stride is 2, the size is decreased by 2. The cells have been integrated from an optimizing method. The network progress is concentrated on 3 features: the cell infrastructure, the amount of cells that are stacked (*N*), and the amount of filters from the primary layer (*F*). Primarily *N* and *F* are set in the search. Then, *N* and *F* from the primary layer are changed for controlling the depth as well as the width of networks. If the search was complete, methods are created with various sizes for fitting the data set. The cell is then related in an optimizing method for developing the NASNet infrastructure. All the cells are associated with 2 input states named hidden state. For providing higher accuracy, NASNetLarge is obtained *N* as 6, but the essential concern to NASNetMobile is for running with restricted resources. In order to both normal as well as reduce cells, an input size of 224 × 224 × 3 was decreased to a size of 7 × 7 at the output with a chosen group of functions utilizing 5B cells. A novel model named scheduled DropPath was presented in NASNet, whereas all the paths from the cell were dropped with linearly enhancing probability as trained of network progress.

### 2.3. Image Classification: DBN Model

During image classification process, the DBN model allocates proper class labels to it. DBN is a probabilistic generation model comprising a stack of restricted Boltzmann machine (RBM) and backpropagation (BP) neural networks. It encompasses the visible layer, *n* hidden, and output layers [20]. The input/visible layer is placed at the end of the model, and the features are passed via many hidden layers at the time of the learning procedure. At last, the proper class label will be allocated at the output layer. In addition, RBM comprises input and hidden layers where bidirectional links exist among two layers. Consider that there are *m* units in the input layer with vector *v*={*v*_1_, *v*_2_, ⋯, *v*_*i*_,   ⋯ *v*_*m*_} and *n* units in the hidden layer with vector *h*={*h*_1_, *h*_2_, ⋯*h*_*n*_}. The energy function of the RBM can be represented using the following equation:

(4) $$\begin{array}{c} E\left(v,\;h;\theta \right)=-\sum_{i=1}^{m}\sum_{j=1}^{n}\omega_{ij}v_{i}h_{j}-\sum_{i=1}^{m}a_{i}v_{i}-\sum_{j=1}^{n}b_{j}h_{j}, \end{array}$$

where *θ* signifies the parameters of RBM, comprising unit bias of input layer *a*_*i*_ and unit bias of hidden layer *b*_*i*_, and *ω*_*ij*_ denotes link weight among the nodes that exist among the input and hidden layers. Based on the energy function of the RBM model, the joint distribution can be defined as follows:

(5) $$\begin{array}{c} p\left(v,\;h\right)=\frac{1}{R\left(\theta \right)}e^{-E\left(v,h\right)},\\ R\left(\theta \right)=\sum_{v,h}e^{-E\left(v,h\right)}, \end{array}$$

where *R*(*θ*) is termed as a normalization factor. The independent probability distribution of the input layer can be formulated as follows:

(6) $$\begin{array}{c} p\left(v\right)=\sum_{h}p\left(v,\;h\right)=\frac{1}{R\left(\theta \right)}\sum_{h}e^{-E\left(v,h\right)}. \end{array}$$

As there exist no links among the nodes in the equivalent layer, the conditional probability distribution of all layers can be defined as follows:

(7) $$\begin{array}{c} p\left(h_{j}=1|v;\theta \right)=\sigma \left(\sum_{i=1}^{m}\omega_{ij}v_{j}+b_{j}\right),\\ p\left(v_{i}=1|h;\theta \right)=\sigma \left(\sum_{j=1}^{n}\omega_{ij}h_{j}+a_{i}\right), \end{array}$$

where *σ*(*x*)=1/(1+exp (*x*)) indicates sigmoid function. The intention of RBM is the maximization of probability *p*(*v*) via modifying bias *a*_*i*_, *b*_*j*_, and weight *ω*_*ij*_. The RBM parameters set *θ*={*a*_*i*_, *b*_*i*_, *ω*_*ii*_} is attained from training data by the use of the maximum likelihood estimation approach. The gradient value of the parameters can be represented as follows:

(8) $$\begin{array}{c} \frac{\partial \ln p\left(v\right)}{\partial \omega_{ij}}={\langle v_{i}h_{j}\rangle }_{\text{data}}-{\langle v_{ij}h\rangle }_{\text{model}},\\ \frac{\partial \ln p\left(v\right)}{\partial a_{i}}={\langle v_{i}\rangle }_{\text{data}}-{\langle v_{i}\rangle }_{\text{model}},\\ \frac{\partial \ln p\left(v\right)}{\partial b_{j}}={\langle h_{j}\rangle }_{\text{data}}-{\langle h\rangle }_{\text{model}}, \end{array}$$

where 〈·〉_data_ signifies the probability of *p*(*hv*) derived by RBM, 〈·〉_model_ characterizes probability *p*(*v*, *h*) provided by the reconstructed RBM. Also, the parameter set *θ* can be reorganized using the contrast divergence model.

(9) $$\begin{array}{c} \omega_{ij}^{\left(t+\Delta t\right)}=\omega_{ij}^{\left(t\right)}+\frac{\alpha }{\beta }\left({\langle v_{i}h_{j}\rangle }_{\text{data}}-{\langle V_{i}h_{j}\rangle }_{\text{model}}\right),\\ a_{i}\left(\left(=a_{j}+\frac{\alpha }{\beta }\left({\langle v_{j}\rangle }_{\text{data}}-{\langle v_{j}\rangle }_{\text{mode}1}\right)\right.\right.,\\ b_{j}^{\left(t+\Delta t\right)}=b_{j}^{\left(t\right)}+\frac{\alpha }{\beta }\left({\langle h_{j}\rangle }_{\text{data}}-{\langle h_{j}\rangle }_{\text{model}}\right), \end{array}$$

where *α* and *β* indicate learning rate and batch size. Once the initial training process of RBM is done, the present hidden layer turned it into the visible layer of the succeeding RBM. Once every RBM training is done, the deep features are classified.

### 2.4. Hyperparameter Optimization: EGOA Algorithm

The hyperparameter tuning of the DBN model is performed using the EGOA algorithm which in turn boosts the classification outcomes. GOA emulates the behavior of grasshopper insects. This insect affects agriculture and crop productivity, and the life cycle comprises egg, nymph, and adulthood [21]. In the nymph stage, the key feature includes moving and jumping in the rolling cylinder (with slow movement and small steps). In the adulthood stage, grasshopper migrates a longer distance in a swarm (with long-range and abrupt movement). Such behaviors are arithmetically expressed by taking the location of the grasshopper into account (*x*_*i*_).

(10) $$\begin{array}{c} x_{i}=S_{i}+G_{i}+A_{i},\;i=1,2,\ldots ,N, \end{array}$$

whereas *S*_*i*_ signifies social interaction of the ith grasshopper as follows:

(11) $$\begin{array}{c} S_{i}=\sum_{j=1,i\neq j}^{N}s\left(d_{ij}\right)\hat{d_{ij}},\;d_{ij}=\left|x_{i}-x_{j}\right|. \end{array}$$

Now, *d*_*ij*_ indicates the distance between the *i*th and *j*th grasshoppers whereas *s* denotes the strength of social force function.

(12) $$\begin{array}{c} s\left(y\right)=fe^{-y/1}-e^{-y}. \end{array}$$

In which *G*_*i*_ and *A*_*i*_ represents the gravity force and wind advection for *i*th grasshopper correspondingly, *l* and *f* indicate the attractive length scale and the intensity of attraction as follows:

(13) $$\begin{array}{c} G_{i}=-g{\hat{e}}_{g},\\ A_{i}=u{\hat{e}}_{w}, \end{array}$$

where *e*_*w*_ and *e*_*g*_ represent the unity vector to the direction of the wind and the center of Earth, and *g* and *u* represent the gravitational constant and constant drift correspondingly. But equation (10) could be directly used for finding the solution to the optimization issue; hence, the researcher is rewritten as the following equation:

(14) $$\begin{array}{c} x_{i}=c\left(\sum_{j=1,i\neq j}^{n}c\frac{u-1}{2}s\left(\left|x_{j}-x_{i}\right|\right)\frac{x_{j}-x_{i}}{d_{ij}}\right)+\hat{T_{d}}, \end{array}$$

where *l* and *u* represent the lower and upper bounds of the searching region, correspondingly; *T*_*d*_ denotes the value of the optimal solution, and *s* is determined in equation (12). But, in equation (14), gravity is not taken into account, and the direction of the wind is often considered as ${\hat{T}}_{d}$. Now, *c* represents a reduction coefficient to shrink the attraction, comfort, and repulsion zones.

(15) $$\begin{array}{c} c=c_{\;\max\;}-t\frac{c_{\;\max\;}-c_{\;\min\;}}{t_{\;\max\;}}, \end{array}$$

where *c*_ max _ and *c*_ min _ represent the maximal value (equivalent to 1) and minimal value (equivalent to 0.00001) of *c*, correspondingly; *t* denotes the existing iteration, and *t*_ max _ represent the maximal amount of iterations. At last, the pseudocode of the GOA is given in Algorithm 1.

In the EGOA, the OBL approach was utilized for determining the opposite solution to the existing solution, and it then utilizes the value of fitness function (*f*) for determining if the opposite has superior to the existing solutions. The fundamental explanation of OBL is presented in [22], by considering the opposite value $\bar{x}$ to the real value *x* ∈ [*u* that is computed as

(16) $$\begin{array}{c} \bar{x}=u+l-x. \end{array}$$

This definition is the generalization to *n*‐dimensional by utilizing the following subsequent formula:

(17) $$\begin{array}{c} \bar{x}=u_{i}+l_{i}-x_{i},\;i=1,2,\ldots ,N, \end{array}$$

whereas $\bar{x}\in R^{n}$ refers to the opposite vector in the real vector *x* ∈ *R*^*n*^. Besides, with the optimized procedure, the 2 solutions (*x* and $\left.\bar{x}\right)$ are calculated, and the optimum solution is saved, but the other was eliminated by relating the fitness function. For sample, if $f\left(x\right)\underline{<}f\left(\bar{x}\right)$ (to minimized), *x* is stored; else, $\bar{x}$ is saved.

## 3. Results and Discussion

This section investigates the oral cancer classification performance of the IDL-OSCDC model using the benchmark Kaggle repository [23]. The dataset includes images of lips and tongue which are classified into cancerous and noncancerous groups. A sample image is demonstrated in Figure 3.

Figure 4 showcases various confusion matrices created by the IDL-OSCDC model on distinct sets of TR/TS datasets. On the training/testing (TR/TS) set of 90 : 10, the IDL-OSCDC model categorized 9 samples into cancer and 4 samples into noncancer. In line with the TR/TS set of 80 : 20, the IDL-OSCDC technique has categorized 18 samples into cancer and 7 samples into noncancer. Meanwhile, on the TR/TS set of 70 : 30, the IDL-OSCDC approach has categorized 24 samples into cancer and 14 samples into noncancer. Eventually, on the TR/TS set of 60 : 40, the IDL-OSCDC system has categorized 28 samples into cancer and 22 samples into noncancer.

Table 1 and Figure 5 report an extensive oral cancer classification performance of the IDL-OSCDC approach on the test and training dataset. The results are inspected under distinct sizes of TR/TS data. The experimental outcome signified that the IDL-OSCDC model has reached proficient values under all sizes of TR/TS data. For instance, with TR/TS set of 90 : 10, the IDL-OSCDC model has provided accu_*y*_, prec_*n*_, reca_*l*_, and *F*_score_ of 92.86%, 90%, 95%, and 91.81%, respectively.

Following this, with a TR/TS set of 80 : 20, the IDL-OSCDC methodology has offered accu_*y*_, prec_*n*_, reca_*l*_, and *F*_score_ of 92.59%, 88.89%, 95%, and 91.12% correspondingly. Along with that, with TR/TS set of 70 : 30, the IDL-OSCDC model has given accu_*y*_, prec_*n*_, reca_*l*_, and *F*_score_ of 95%, 96.15%, 93.75%, and 94.67% correspondingly. Furthermore, with TR/TS set of 60 : 40, the IDL-OSCDC method has provided accu_*y*_, prec_*n*_, reca_*l*_, and *F*_score_ of 94.34%, 94.11%, 94.49%, and 94.27% correspondingly.

A brief precision-recall examination of the IDL-OSCDC model on different TR/TS datasets is portrayed in Figure 6. By observing the figure, it is noticed that the IDL-OSCDC model has accomplished maximum precision-recall performance under all datasets.

Figure 7 demonstrates the ROC inspection of the IDL-OSCDC model under different sets of training and testing datasets. The result indicates that the IDL-OSCDC model has resulted in the highest performance on the testing dataset over the other ones.

Figure 8 illustrates the training and validation accuracy investigation of the IDL-OSCDC approach on the applied dataset. The figure conveyed that the IDL-OSCDC model has offered maximum training/validation accuracy in the classification process.

Next, Figure 9 represents the training and validation loss examination of the IDL-OSCDC model on the applied dataset. The figure reported that the IDL-OSCDC model has exhibited reduced loss values.

Table 2 investigates the comparative study of the IDL-OSCDC technique with recent approaches [24].  Figure 10 inspects the detailed accu_*y*_ examination of the IDL-OSCDC model with other models. The figure revealed that the SVM method has resulted in least performance with a lower accu_*y*_ of 88.38%. In addition, the ANN-SVM technique has reached a slightly enhanced outcome with accu_*y*_ of 90.48% whereas the fuzzy technique has depicted a moderately improved accu_*y*_ of 92.76%. Following this, the RF and CapsNet technique have shown closer results than the other methods. However, the IDL-OSCDC model has shown an effectual outcome with a maximum accu_*y*_ of 95%.

Figure 11 examines the detailed prec_*n*_, reca_*l*_, and *F*_measure_ examination of the IDL-OSCDC model with other techniques. The figure exposed that the SVM system has resulted in least performance with lower prec_*n*_, reca_*l*_, and *F*_measure_ of 89.82%, 90.65%, and 88.01%. Furthermore, the ANN-SVM model has reached slightly enhanced outcome with prec_*n*_, reca_*l*_, and *F*_measure_ of 92.24%, 90.13%, and 91.94% whereas the fuzzy method has portrayed moderately enhanced prec_*n*_, reca_*l*_, and *F*_measure_ of 88.03%, 89.43%, and 91.53%. Afterward, the RF and CapsNet models have revealed closer results over the other methods. Finally, the IDL-OSCDC algorithm has shown effectual outcome with maximum prec_*n*_, reca_*l*_, and *F*_measure_ of 96.15%, 93.75%, and 94.67%. After observing the abovementioned figures and tables, it is apparent that the IDL-OSCDC model has resulted in maximum performance over the other methods.

## 4. Conclusion

In this article, a novel IDL-OSCDC model has been established for the identification and classification of oral lesions using biomedical images. At the initial stage, the IDL-OSCDC model utilized the GF technique to get rid of noise content. Following this, the NasNet model is exploited for the generation of higher-level deep features from the input images. Finally, the EGOA-DBN model is utilized to detect and categorize oral cancer. The hyperparameter tuning of the DBN model is performed using the EGOA algorithm which in turn boosts the classification outcomes. The experimentation outcomes of the IDL-OSCDC model are performed using a benchmark biomedical imaging dataset. An extensive comparison study highlighted its promising performance over the other methods. In the future, advanced DL models can be utilized as a classifier to optimize the detection performance.

## Figures and Tables

**Figure 1:** Overall process of IDL-OSCDC technique.

**Figure 2:** Structure of NASNet model.

**Figure 3:** Sample images.

**Figure 4:** Confusion matrix of IDL-OSCDC technique with different TR/TS datasets.

**Figure 5:** Overall result analysis of IDL-OSCDC technique.

**Figure 6:** Precision-recall analysis of IDL-OSCDC technique with diverse TR/TS datasets.

**Figure 7:** ROC analysis of IDL-OSCDC technique with different TR/TS datasets.

**Figure 8:** Accuracy graph analysis of IDL-OSCDC technique.

**Figure 9:** Loss graph analysis of IDL-OSCDC technique.

**Figure 10:** Acc_*y*_ analysis of IDL-OSCDC method with current algorithms.

**Figure 11:** Comparative analysis of IDL-OSCDC approach with recent algorithms.

**Algorithm 1:** Pseudo-code of GOA

**Table 1:** Classification results of IDL-OSCDC technique on TR/TS datasets.

Class labels	Accuracy	Precision	Recall	F-score
Training/Testing (90 : 10)				
Cancer	92.86	100.00	90.00	94.74
Noncancer	92.86	80.00	100.00	88.89
Average	92.86	90.00	95.00	91.81

Training/Testing (80 : 20)				
Cancer	92.59	100.00	90.00	94.74
Noncancer	92.59	77.78	100.00	87.50
Average	92.59	88.89	95.00	91.12

Training/Testing (70 : 30)				
Cancer	95.00	92.31	100.00	96.00
Noncancer	95.00	100.00	87.50	93.33
Average	95.00	96.15	93.75	94.67

Training/Testing (60 : 40)				
Cancer	94.34	96.55	93.33	94.92
Noncancer	94.34	91.67	95.65	93.62
Average	94.34	94.11	94.49	94.27

**Table 2:** Comparative analysis of IDL-OSCDC approach with recent algorithms.

Method	Accuracy	Precision	Recall	*F*-measure
SVM model	88.38	89.82	90.65	88.01
Fuzzy technique	92.76	88.03	89.43	91.53
ANN-SVM model	90.48	92.24	90.13	91.94
RF model	94.78	88.50	92.06	88.95
Capsule network model	94.35	95.90	92.78	93.33
IDL-OSCDC	95.00	96.15	93.75	94.67

## Data Availability

Data sharing is not applicable to this article as no datasets were generated during the current study.
